This article has been retracted.

# Construction of a Digital Elderly Care Service System Based on Human-Computer Interaction from the Perspective of Smart Elderly Care

**DOI:** 10.1155/2022/1500339

**Published:** 2022-05-20

**Authors:** Yifei Zhou

**Affiliations:** School of Public Administration, Zhongnan University of Economics and Law, Wuhan 430000, Hubei, China

## Abstract

Digital elderly care service is an innovative elderly care model, and its emergence has brought about a huge change in the field of elderly care services (ECSS). The current method is to make the elderly care service more precise and personalized, improve the ability and level, and improve the current ECSS. The defect is that the short of top-level design and overall planning is basically only in the state of trial operation. In order to solve these problems, this paper proposes to study how to intervene in social work in smart ECSS to enhance service capabilities and improve service quality on the original basis. Therefore, based on the use of human-computer interaction technology, this paper deepens the research on the current elderly care services. According to a survey of the elderly in a certain city, the digital elderly care system shows that 25.33% of the elderly prefer to use housekeeping services, and 63% of the elderly prefer healthcare services. The results show that the digital elderly care service system based on human-computer interaction technology is easier to be accepted by the elderly than the traditional elderly care service. The elderly care service system under human-computer interaction is more considerate than the traditional elderly care service system and can make the elderly's life more colorful.

## 1. Introduction

### 1.1. Background

In recent years, the problem of aging and null nesting in China has become more and more serious. At this stage and in the future, people will have to face the problem of old-age care that needs to be solved urgently. Affected by various factors such as population, family structure, China's urbanization process, and traditional concepts, the community, as the basic unit of residents' life, will provide people with comprehensive and systematic elderly care services. With the proposal of the concept of “smart elderly care,” people began to consider using advanced human-computer interaction technology to serve the community, realize the effective integration of elderly care service resources, and provide better services for the elderly. The smart community elderly care service management system combines traditional community elderly care service stations with today's big data Internet to realize all the processes of the elderly from needing to solving needs. Whether it is the elderly's personal safety issues, medical issues, daily needs, or the elderly's usual activities and hobbies, there is a complete management system, which can clearly record the massage of the elderly and remind the elderly to pay attention in time. Besides, the management of information files of the elderly by government departments has become more convenient and organized. The smart community elderly care service management system is committed to scientifically manage the diet and everyday life of the elderly, so that the elderly can get the best elderly life without the constraints of time and space.

### 1.2. Significance

Under the case of aging in China, community pension emerges as a new way of pension, integrating benefits of family pensions and organizational pensions, and concentrated pension services in the community. The elderly still live in a familiar environment, and they communicate with familiar friends, which not only respects the traditional concepts of the elderly, but also facilitates the care of children in their spare time. It can also fully integrate and utilize the resources of families and communities to offer professional services for the elderly and reduce the cost of old-age care. This is a universal pension method that adapts to the growth of China's national conditions.

### 1.3. Innovation

The innovations of this paper are as follows: (1) first of all, the elderly do not have to leave their original living environment and social relations to enjoy services for the elderly at home, so that the feelings and needs of the elderly can be respected. (2) Secondly, take the elderly as the center and make full use of the resources of family, community and society, so as to greatly reduce the cost of old-age care. Through the informatization of smart elderly care services, the government, individuals, families, institutions, and operators are connected to achieve full information interconnection, give full play to the efficiency of resources, and improve the life and quality of life of the elderly. (3) Finally, the comprehensive construction of smart community elderly care services will be of great benefit to accelerating the development of the service industry, increasing jobs, and achieving economic growth in the service industry.

## 2. Related Work

Mukherjee et al. believe that human-computer interaction can automatically predict regular activities, walking, running, cooking, performing office work, etc. as an example in daily life. It is really nice in the field of artificial intelligence, healthcare services such as personal healthcare assistants, aged care services, maintaining patient records for future help, etc. [1]. Zhang et al. also believe that the human-computer interaction problem of each component of the smart elderly care service ecosystem is how to deal with the interest relationship between multiple resource subjects [2]. Tai et al. proposed a human-computer interaction system applied to the motion model of the elderly, which can transmit the positioning data set in real time when a fall occurs, so that the treatment can be carried out quickly and properly, and the injury caused by the fall to the elderly can be minimized [3]. Zhou et al. showed that using the theory and principles of human-computer interaction can help the adoption of smart elderly care to be selected as a decision-making attribute. The remaining attributes are used as conditional attributes and multi-level symmetric attribute sets to evaluate the acceptance of smart old age care [4]. Yi et al. explored and analyzed an interactive home care 2-way video health care system. Through research and interviews, they analyze the day-to-day life and behaviors of the elderly in their homes, obtain the primary requirements of the elderly in their lives, as well as their cognitive and behavioral characteristics, and construct an ECSS for the elderly [5]. According to Yang et al., smart home care has drawn a lot of study attention recently and remains an active problem. IoT has been identified as a critical enabler for enabling smart home care [6]. Zhu et al. proposed that the strategy of service offering and reimbursement of the combined medical and health care model should be adjusted to improve the health protection level of the elderly and promote health equity, for one thing, with the goal of strengthening the service supply of combined medical and health care, guiding the elderly to reasonably choose the combined medical and health care model, and paying attention to the spiritual and cultural needs of the elderly and end-of-life care [7]. Hu et al. proposed a telemedicine service system. Based on human-computer interaction technology, the system collects real-life data through an environmental sensor package (including binary motion, contact, pressure, and proximity sensors) installed in the homes of the elderly [8]. However, these studies are not practical enough.

## 3. Human-Computer Interaction Technology

### 3.1. Human-Computer Interaction

Human-computer interaction technology refers to the technology that realizes the dialogue between human and computer in an effective way through computer input and output devices. Human-computer interaction technology includes that machines provide a large amount of relevant information and prompt requests to humans through output or display devices, and people input relevant information to machines through input devices, answer questions, and prompt requests for instructions. Human-computer interaction technology is one of the important contents in computer user interface design. Human-computer interaction technology is one of the fastest-growing fields in user interface research, and all countries attach great importance to it. Among the national key technologies in the United States, the human-machine interface is listed as one of the six key technologies in information technology, along with software and computers, and it is called “it has outstanding importance to the computer industry and is also very important to other industries.”

### 3.2. Somatosensory Technology

Somatosensory technology is a technology that allows people to interact with content without the use of any complex control devices. The human-computer interaction process based on somatosensory devices is shown in Figure 1:

Compared with physical interaction methods such as voice and limbs, the advantages of gesture interaction are obvious. First of all, the way of viewing interaction is more intuitive and easy to understand than others. Operators can directly express their operational intentions, and secondly it is the most versatile.

#### 3.2.1. Application of Somatosensory Kinect

Kinect somatosensory has good characteristics in bone tracking and speech recognition and is widely used in space exploration, commerce, medicine, robotics, and computers. Figures 2 and 3 are the Kinect somatosensory.

Its main technical parameters are shown in Table 1:

#### 3.2.2. Kinect R&D Introduction

From version 1.8 of Kinect SDK, it can be seen that the API includes three components: NUI API, Kinect Audio DMO, and Window Speech SDK. Among them, NUI API is the core component of Kinect SDK. Its API stack is shown in Figure 4:

#### 3.2.3. Kinect Depth Image Imaging Principle

Kinect obtains the depth value of objects in the scene through triangulation and takes the center *A* of the infrared camera as the origin, and the direction of the *x*-axis points from the origin *A* to the infrared projector *B*. The *z*-axis represents the gray value of the pixels in the image [9]. Among them, *Z*_0_ is the depth value of the reference plane; when the object plane does not coincide with the reference plane, the position of the speckle pattern will be offset, and e is the offset; *m* is the distance between the infrared camera and the infrared projector; *f* is the focal length of the infrared camera; *E* is the distance between the target point *i* and the reference point *o*, so we have

(1) $$\begin{array}{c} \frac{E}{M}=\frac{E_{0}-Z_{i}}{Z_{0}}, \end{array}$$

(2) $$\begin{array}{c} \frac{e}{m}=\frac{E}{Z_{i}}. \end{array}$$

By combining formulas (1) and (2), the depth value of the target point *i* can be obtained:

(3) $$\begin{array}{c} Z_{a}=\frac{Z_{0}}{1+Z_{0}/\text{lm}\;e}. \end{array}$$

#### 3.2.4. Kinect Data Structure

With the development of computer vision technology, the technology of obtaining 3D data on the surface of objects in the scene through depth image data has become more and more mature, and depth images are different from 2D images [10].

#### 3.2.5. Depth Image Data Flow

Kinect generates a stream of depth image data at 30 frames per second, occupying 2 bytes per pixel. In fact, the depth image captured by Kinect only occupies one byte. In order to meet the storage requirement of 2 bytes, the depth value needs to be further processed. The depth value is located in the upper 13 bits, so it needs to be shifted to the right by 3 bits to obtain the depth value of the changed pixel, and then the gray value can be calculated by the following formula:

(4) $$\begin{array}{c} Z_{i}=255-\left(\frac{256*D_{i}}{4095}\right). \end{array}$$

Among them, *Z*_*i*_ represents the gray value of pixel *i*, *D*_*i*_ represents the depth value of pixel *i*, and its value range is 0–4095. It can be known from the formula that the gray value is determined by the depth value, and the larger the depth value is, the smaller the gray value is. The depth value reflects the distance between the object and the camera. The closer the distance between the two, the smaller the depth value, and the higher the gray value.

#### 3.2.6. Somatosensory Sensor Leap Motion

Leap Motion is a somatosensory controller developed by the American company LEAP in 2012 to recognize human hands. Its structure is shown in Figure 5.

Leap Motion's components consist primarily of filters, 2 high frame-rate infrared cameras, 3 infrared LEDs, and a chip. The infrared cameras capture information about the movement of a person's hand in 3D space, while the infrared LEDs are used to improve lighting conditions.

#### 3.2.7. Working Principle of Leap Motion

Leap Motion employs dual vision stereo localization technology to capture hand motion information. When Leap Motion picks up a hand gesture, a strainer first filters ambient daylight to obtain infrared light and creates a grid of infrared light above it. When a person's hand appears in the recognition area over it, the infrared light is reflected, and the camera captures a high-definition image of the person's hand and then obtains 3D data information about the person's hand through binocular stereo vision. This method is commonly used for spatial object localization.

### 3.3. Target Recognition and Tracking Based on Kinect

Target recognition and tracking mainly includes the identification of target personnel and the location tracking of target personnel. The following shows the whole process of target recognition and tracking, as shown in Figure 6.

#### 3.3.1. Target Person Recognition Based on Color Histogram Matching

In this paper, Kinect is used to identify and track the target person in the scene. When multiple targets appear in the work area at the same time, it is required to be able to quickly and accurately identify the designated person and track the location, but not to identify the nontarget person, which involves the problem of identification. Since the Kinect SDK does not have an identity recognition function, a person recognition method based on image information is adopted. The color image of the scene is captured by Kinect, and then the target person in the scene is identified according to the color histogram matching result [11]. The color histogram is mainly used to describe the proportion of different colors in the whole image. Commonly used color histogram matching methods mainly include correlation chi-square and intersection. The relevant calculation formulas are as follows:

(5) $$\begin{array}{c} d_{\text{dreep}}\left(H_{1},H_{2}\right)=\frac{\sum_{i}H_{1}\left(i\right)H_{2}\left(i\right)}{\sqrt{\sum_{i}H_{1}^{2}\left(i\right)H_{2}^{2}\left(i\right)}},\\ H_{k}^{\prime }\left(i\right)=H_{k}\left(i\right)-\frac{1}{N}\left(\sum_{J}H_{k}\left(j\right)\right). \end{array}$$

Among them, *N* represents the equal number of *H* components, and *H*_1_, *H*_2_ are the histogram functions. The formula for calculating chi-square is as follows:

(6) $$\begin{array}{c} d_{\text{chips}}\left(H_{1},H_{2}\right)=\sum_{i}\frac{{\left(H_{1}\left(i\right)-H_{2}\left(i\right)\right.}^{2}}{H_{1}\left(i\right)+H_{2}\left(i\right)}. \end{array}$$

It can be obtained from the above that

(7) $$\begin{array}{c} d_{\text{intersection}}\left(H_{1}\right)\left(H_{2}\right)=\min\sum_{i}H_{1}\left(i\right)H_{2}\left(i\right). \end{array}$$

According to the above formula, the matching result reference table shown in Table 2 is obtained.

It can be seen from Table 2 that the larger the calculation result of the correlation and intersection matching algorithm, the higher the matching degree of its histogram, and its value is 1 when it is completely matched. The smaller the calculation result of the chi-square matching algorithm, the higher the matching degree of its histogram, and the value is 0 when it is completely matched.

#### 3.3.2. Gesture Data Processing Based on Kalman Filtering

In order to eliminate the influence of human handshake and environmental factors on gesture data, the Kalman filter algorithm is used in this paper to iteratively calculate the optimal value and measured value of gesture data to eliminate the noise introduced by human handshake and environmental factors. Kalman filtering is also known as the optimal estimation method, which can estimate the optimal value of the dynamic system in the next period according to the data with noise. In the prediction stage, the predicted value in the current state and the certainty of the predicted value are obtained by calculation. In the update stage, the predicted value is updated to the optimal value according to the weight, and the certainty of the optimal value is calculated. The weights are calculated from a series of data and predicted values, and their magnitudes are determined by certainty [12]. Finally, the predicted value of the next stage is calculated according to the optimal value and certainty in the current state. Due to the recursive nature of the Kalman filtering algorithm, the optimal value of the current state can be accurately calculated only according to the measured value of the current state and the optimal value of the previous moment during gesture data processing. The processing efficiency of gesture data and the real-time performance of the system are improved.

Since the Kalman filtering algorithm is calculated on a dynamic system based on the time domain, a discrete control system needs to be introduced, which is represented by the following formula:

(8) $$\begin{array}{c} e_{k+1}=E_{k+1}X_{k}+Q_{k+1}+P_{k+1}. \end{array}$$

Among them, *e*_*k*+1_ represents the system state at time *k* + 1; *X*_*k*_ represents the system state at time *k*; *E*_*k*+1_ represents the transformation matrix acting on *X*_*k*_; *Q*_*k*+1_ represents the control parameter; *V*_*k*+1_ is the control matrix. When *V*_*k*+1_ = 0, the system has no control parameters; *P*_*k*+1_ is the system noise, which obeys the normal distribution *P*_*k*+1_∼*N* (0, *y*_*k*+1_).

At time *k* + 1, the measured value *L*_*k*+1_ satisfies the following formula:

(9) $$\begin{array}{c} L_{k+1}=H_{K+1}x_{k+1}+v_{k+1}. \end{array}$$

Among them, *H*_*k*+1_ is the measurement matrix that projects the state of the system at time *x*_*k*+1_ to the measurement space; *v*_*k*+1_ is the measurement noise.

The calculation assumes that the initial state *x*_0_, system noise, and measurement noise are independent. According to the formula, the state value at time *k* + 1 can be obtained:

(10) $$\begin{array}{c} x\left(k+1|k\right)=F_{k+1}x\left(k|k\right)+T_{k+1}v\left(k+1\right). \end{array}$$

Among them, *x*(*k*+1*|k*) represents the prediction of the optimal numerical at time *k* + 1 by the state numerical of the system at time *k*+1 represents the optimal numerical at time *k*; *x*(*k|k*) is the control amount of the system at time *k* + 1. In this paper, the numerical of *v*(*k*+1) is 0, so the formula can be simplified as

(11) $$\begin{array}{c} x\left(k+1|k\right)=F_{k+1}x\left(k|k\right). \end{array}$$

In the Kalman filter prediction stage, the position and attitude information is obtained by calling the Leap SDK, and then the predicted value of the position and attitude of the human hand at the next moment is predicted according to the Kalman filter algorithm. Assuming that, at time *k*, the position coordinate of the palm is *O*_*k*_, and the velocity and acceleration are *v*_*k*_, *a*_*k*_ respectively, then according to the law of motion,

(12) $$\begin{array}{c} s=v_{k}t+\frac{1}{2}a_{k}t^{2},\\ Q_{k+1}=Q_{k}+s. \end{array}$$

Among them, *p*_*k*+1_ is the position coordinate of the hand at time *t*. In the update stage of Kalman filtering, the position deviation *p k k* (1) is first updated as follows:

(13) $$\begin{array}{c} Q_{k+1}=F_{k+1}Q\left(k|k\right)F_{k+1}^{\prime }+r. \end{array}$$

Among them, *p*(*k|k*) indicates that the deviation value of *x* (*k|k*) at time *k* is the transpose of *F*_*k*+1_, and *r* is the system deviation.

The predicted value at time *k* + 1 is obtained by calculation, and the measured value at time *k* + 1 is obtained by the sensor, and then the optimal value at time *k* + 1 is

(14) $$\begin{array}{c} x\left(k+1|k+1\right)=x\left(k+1|k\right)+c\left(k+1\right)*\left(Z\left(k+1\right)-h\right)\left(k+1|k\right). \end{array}$$

Among them, *c* (*k* + 1) is the Kalman gain at time *k* + 1, and its expression is

(15) $$\begin{array}{c} c\left(k+1\right)=\frac{\left(k+1|k\right)H{}^{\prime }}{\left(H_{p}\left(k+1|k\right)H{}^{\prime }\right)+r}. \end{array}$$

At time *k* + 1, the deviation value of *x*(*k*+1*|k*+1) is

(16) $$\begin{array}{c} p\left(k+1|k+1\right)=\left(1-c\right)k\left(H\right)p\left(k+1|k\right). \end{array}$$

Through recursive calculation, the optimal value *x*(*k*+2*|k*+2) and the deviation value *p*(*k*+2*|k*+2) at time *k* + 2 can be obtained, and by analogy, continuous gesture information can be obtained.

#### 3.3.3. Finger Kinematics Model

In order to obtain more detailed gesture information, it is necessary to obtain the state information of each joint of the finger by constructing a kinematic model of the finger. From the perspective of human hand anatomy, it is generally believed that the fingers include the distal phalanx, the middle phalanx, the proximal phalanx, and the four segments of the metacarpal. They are connected by three joints: the distal finger joint (DIP), the proximal finger joint (PIP), and the metacarpophalangeal joint (MCP). From the kinematics point of view, both the distal and proximal finger joints have only 1 degree of freedom, and the metacarpophalangeal joint has 2 degrees of freedom. When recognizing the grasping action of the human hand, the longitudinal motion of each joint is mainly recognized. Therefore, in order to reduce the influence of human hand shake on gesture recognition accuracy, the final finger model only contains 3 joints of each finger [13]. The spatial coordinates of each joint of the finger and the direction vector of the finger can be obtained through Leap SDK, and the corresponding joint angle can be obtained according to the direction vector between two adjacent phalanges. As shown in Figure 7, three joint points constitute a finger plane, *θ*_1_, *θ*_2_, *θ*_3_ and *ℓ*_1_, *ℓ*_2_, *ℓ*_3_, *ℓ*_4_ are the joint angle and the direction vector of each segment of the phalanx, respectively. Among them, *θ*_2_ and *θ*_3_ can be obtained according to the direction vectors of adjacent joints, and the rest only need to solve *θ*_1_. Figure 7 shows the finger kinematics model.

*θ*_1_ is the angle between the metacarpal bone and the proximal phalanx. Considering that the plane of the metacarpal bone coincides with the plane of the palm, *θ*_1_ can be regarded as the angle between the plane of the proximal phalanx and the plane of the palm, and *θ*_1_ is 0 when the finger is straight. Let the normal vector of the intersection of the palm plane and the proximal phalanx plane be *ℓ*_5_, and then there is *θ*_1_:

(17) $$\begin{array}{c} \ell_{5}=n_{1}*n_{2}. \end{array}$$

In the formula, *n*_1_ is the normal vector of the finger plane.

(18) $$\begin{array}{c} n_{1}=\ell_{1}*\ell_{2}. \end{array}$$

*n*_2_ is the normal vector of the palm plane.

Then, the expression for *θ*_1_ is

(19) $$\begin{array}{c} \theta_{1}=\text{arccos}\left(\ell_{2}*\ell_{5}\right). \end{array}$$

It can be seen from the above that the finger kinematics model is used to build a platform for somatosensory technology; that is, to help the construction of smart community elderly care services based on human-computer interaction is the top priority. Compared with traditional elderly care services, the use of fingers to transmit messages and seek help can enable most elderly people to better obtain high-quality elderly care services.

## 4. Construction of the Elderly ECSS

### 4.1. Design of Pension System

The content of this chapter is mainly to provide a general analysis and explanation of the overall structure of the smart community elderly care service management system, the smart community elderly care service technical architecture, the smart community elderly care service functional architecture, and the smart community elderly care service network architecture. The overall architecture design of the smart community elderly care service management system is shown in Figure 8.

The development language of the smart community pension service management system has chosen the object-oriented development language Java for project development. The framework uses the SSH integration framework and assists the use of the MVC design pattern. The use of layers facilitates the future management and maintenance of the system and reduces the burden of maintenance personnel. The smart community aged care service management system has designed a smart community aged care service management presentation layer, a smart community aged care service management business logic layer, and a smart community aged care service management persistent layer. The presentation layer mainly includes Struts-MVC and AJAX, the business logic layer is mainly responsible for Spring, and the persistence layer is responsible for Hibernate [14].

The contents included in the presentation layer mainly include StrutsAction class, ActionForm class configuration file, Struts-configxml, XmlHttpRequest object, and JSP page. The business logic layer mainly includes Spring transaction processing, business service classes, and Hibernate painting management. The persistence layer contains data sources/connection pools as well as query language support and other Hibernate services. The MVC design pattern generally refers to the Model, the View, and the Control. The use of the three-tier architecture first reduces the dependencies between layers, and can independently develop and maintain each layer, which makes the project structure clearer and improves the security of the system.

### 4.2. System Technical Architecture

The smart community pension service management system uses the Java language in the object-oriented programming language to develop the entire system. On the framework of the system, the SSH integration framework is selected for development and use, and the MVC design pattern and B/S network architecture pattern are assisted.

The technical architecture used by the smart community elderly care service management system is shown in Figure 9.

The advantage of the Java language is that it is a pure object-oriented programming language, which is suitable for any platform to realize one compilation and run everywhere. And the Java language itself provides many built-in class libraries to effectively improve the developer's work efficiency, which is why Java can become the most widely used language. The C/S architecture (client/server) requires users to install the client for use, and each time the system is upgraded, the system needs to be downloaded and installed by the user before it can be used. The B/S architecture is also the browser/server mode in the traditional sense. In the system developed by the B/S architecture, users only need a browser to use, no installation is required, and it is simple and easy to operate. The SSH framework is a typical three-tier framework combination, which reduces the burden on developers. In addition, SSH has good scalability, good maintainability, and excellent decoupling [15]. The powerful tag library of Struts framework can improve development efficiency, and Hibernate's L3 cache can save a lot of time. The Spring framework glues the frameworks together better, and the code structure is clearer. The application of Java language to the construction of the technical architecture diagram of the smart community elderly care service management system can accurately demonstrate the structural rigor and integrity of the system's technical architecture.

### 4.3. System Functional Architecture

The functional architecture diagram of the smart elderly care service management system is shown in Figure 10.

The modules are designed by the smart community elderly care service management system, namely, the basic data of smart community elderly care services, comprehensive business, activities, service work orders, service teams, and applications for the elderly.

#### 4.3.1. Basic Data Management

Safety statistical analysis management is to manage and analyze the subdistrict, community service stations, service businesses, community volunteers, service projects, and service terminals. The basic data management mainly designs seven related functional modules, which are the management of subdistrict jurisdiction, community service stations, service businesses, service personnel, community volunteers, service items, and terminals [16]. Among them, the district management of smart community elderly care services is used to add districts, modify districts, delete districts, and export districts. The functions of service merchant management include adding service merchant information, modifying service merchant information, and deleting merchant information in batches. Service personnel management functions include adding service personnel, modifying service personnel, deleting service personnel information in batches, and querying service personnel information. Community volunteer management functions include adding community volunteer groups, modifying volunteer members, deleting volunteer group information, and exporting volunteer member information. Service item management functions include adding service item information, modifying service item information, and deleting service items in batches. The terminal management function includes functions such as querying terminal information and editing and issuing terminal information.

The functional architecture diagram of basic data management is shown in Figure 11.

#### 4.3.2. Elderly File Management

Comprehensive business management is the management and analysis of the elderly's information files, health files, medication records, physical examination records, medical records, and hobbies. The elderly file management mainly designs eight functional modules. They are the audit management of elderly files, elderly information files, elderly health files, elderly medication records, elderly physical examination records, elderly medical records, elderly hobbies management, and elderly tracking and positioning management functions. The functions of the elderly file audit management design include adding elderly information, batch auditing data, and exporting elderly file data. The functions of the elderly information file management design include querying the elderly to be reviewed, modifying the elderly information, deleting the elderly information, and exporting the elderly information. The function of the management design of the elderly health records is to add the information of the elderly health records [17].

### 4.4. System Network Architecture

The network deployment of the smart community elderly care service management system selects the B/S network architecture to design and implement the smart community elderly care service management system. The B/S network architecture is traditionally called the browser/server model. The difference between it and the C/S network architecture is that one is deployed on the server side and used on the client side, and the other is deployed on the server and used on the browser [18].

Compared with the C/S mode, the system client does not need to be installed by the user, and the browser can access it, which greatly increases the convenience of the system [19], and the system is more interactive. The network architecture design diagram of the smart community elderly care service management system is shown in Figure 12.

### 4.5. Database Table Design

A database is a warehouse that organizes, stores, and manages data according to data structures. It is a collection of large amounts of data stored in the computer for a long time, organized, sharable, and uniformly managed. This section will focus on individual database tables in the smart community elderly care service management system in detail. Due to the limited length of the article, a representative data table will be selected for specific display analysis. The specific data tables involved include the user table, the service provider table, the activity table, the service work order table, and the commodity order table.

The user table saves the date of birth, status, home phone, and moderator of smart community users. The number is the primary key of the user table, the reviewer is the foreign key, the link is the user table, and the content is the user's number. Category 1 is for the elderly with minimum living allowances, 2 for the elderly, and 3 for the lonely and widowed elderly. Gender 1 represents male, and 2 represents female. Status 1 means the audit passed; 2 means the audit failed; 3 means unexamined. The user table is shown in Table 3:

The main fields of the service provider table are merchant code, merchant name, merchant category, business license code, service status, business hours, person in charge, contact number, responsible area, service personnel, etc. Among them, the business code is the primary key of the service provider table, and the areas responsible for the area and the service personnel are connected by the foreign key, which are the area table and the user table, respectively. When the service status is 1, it represents normal service, as shown in Table 4.

The main fields of the event table include event number, event name, event type, holding time, start time, end time, event location, next event, contact number, and status, where the activity number is the primary key of the activity table. When the status is 1, it means that the event has been held, and when the status is 2, it means that the event has not been held. The activity table is shown in Table 5:

The main fields included in the service work order table are the work order number, the elderly person's name, the work order status, the work order level, the service personnel, the county, the street, the community, the contact information of the elderly, the address of the elderly, and service items. The work order number is the primary key of the service work order table, the service personnel is the foreign key, and the connection is the user table. When the status of the work order is 1, it means that the order has been dispatched, and when the status is 2, it means that the order has been received. When the work order level is 1, it means normal, as shown in Table 6:

## 5. Discussion of the Results of the Digital Elderly ECSS

In 2017, the State Council issued the “Thirteenth Five-Year Plan for the Development of National Aged Companies and the Construction of the Elderly Service System,” proposing to implement the “Internet+” elderly care service plan to strengthen community construction and nursing home facilities, integrating and building a community-based home-based elderly care service information platform, call service system, and emergency service mechanism to facilitate nursing home institutions and organizations to provide meals, cleaning, walking, bathing, medical assistance, day care, and other services for the elderly at home. The launch and implementation of a series of civilian nursing services have provided a favorable policy environment for the development of smart elderly care services and smart community nursing services [20]. Since 2000, China has entered an aging society, and the aging process has gradually accelerated. From 2012 to 2017, the proportion of the elderly population with household registration in a certain city increased from 20.3% to 24.5%, an increase of 4.2 percentage points as shown in Figure 13.

In order to cope with the increasingly serious aging problem and the growing demand for elderly care, the elderly care services provided by community service centers must meet the needs of the elderly; social organizations and volunteers for the elderly are encouraged. Design and construction departments should design and arrange living facilities and activity venues suitable for the elderly when building urban and rural public facilities and residential areas [21]. In July 2001, a city launched the “Starlight Plan for Community Elderly Care Services” to provide the elderly with functions such as day care services, nursing, health rehabilitation, sports and leisure, home services, and emergency assistance. The use of the elderly care service system under the smart community is ready for the subsequent aging of the population, and the elderly can take care of their lives in the future smart community.

### 5.1. The Use of the Smart Community Elderly Care Service Platform by the Elderly in a City

In general, the three services of housekeeping, health housekeeping, and medical care are the most used by the elderly, and emotional consultation projects are rarely used by the elderly, and some elderly people have not used the functions in the elderly care service platform.  Figure 14 shows the use of various functions of the smart elderly care platform by the elderly (this question may account for more than 100% of the total number of multiple-choice questions in the questionnaire).

The reasons for this can be summarized in the following points: first, living services, medical care, and health management are the living needs of the elderly. Before the implementation of the smart pension platform, there was a need for pensions. However, due to the lack of a platform for providing services, the emergence of smart community elderly care has alleviated the urgent needs of the elderly for this part of the service, so the elderly use these three services more.

At present, smart care for the elderly in China mainly focuses on basic life services, medical diagnosis and treatment, health care, etc. and does not pay as much attention to emotional companionship and recreational activities for the elderly as the former two. Although community-based smart home care services are mostly based on smart care platforms, they do not pay enough attention to the spiritual aspect of the elderly, and most of the services provided can only meet the basic service needs of the elderly. On the other hand, the elderly are more familiar with the content of life care and medical health and use these functions more frequently [22].

### 5.2. The Demand for Smart Community Elderly Care Services for the Elderly in Different Age Groups in a City

This survey divides the needs of the elderly into two parts: life services and entertainment. The following is an analysis of the needs of elderly people of different ages and physical conditions for the services of the two sectors.

#### 5.2.1. Comparison of Demand for Life Services

Figure 15 shows the demand distribution of the three age groups of the elderly for various service items of life services. Combined with the interviews with the elderly, this conclusion can be drawn: generally speaking, in the section of life services, the elderly have a greater demand for housekeeping services and convenient maintenance. Among them, the elderly people aged 60–70 have a similar demand for housekeeping services and convenient maintenance, and the gap is small. The elderly aged 70–80 have significantly higher needs for domestic services than other services. Due to their relatively long age, this part of the elderly seems to have some difficulty in housework such as housework and going out to buy vegetables, so there is a greater demand for this part. The greater needs of the elderly over the age of 80 focus on the aspect of convenient maintenance. Combined with the interviews, the elderly in this age group do not have high requirements for housekeeping services. Generally, children who regularly organize during vacation can meet the needs of the elderly in terms of laundry, bathing, and housekeeping. What makes it difficult for these elderly people are the daily maintenance matters. The maintenance situation is mostly sudden although it does not constitute an obstacle to the life safety of the elderly, but it will bring inconvenience to the life of the elderly. And because the elderly over 80 years old are older and cannot solve it by themselves, if they wait for the help of their children, the damaged household items or electrical appliances can not be used, which will affect their normal life. Therefore, it is their urgent need to obtain convenient maintenance services through the smart pension platform, as shown in Figure 15.

Among other detailed services, seniors aged 70–80 had more outdoor care needs than seniors in the other two age groups. Although these elderly people are not young, their need to go out has not decreased. Currently, seeking care is emerging as the best way to resolve this conflict of needs. Providing volunteers to accompany them to participate in outreach activities, and some elderly people who need help with rehabilitation training due to illness will also have better opportunities for outings and sports.

#### 5.2.2. Comparison of Demand for Recreational Activities

Figure 16 is a comparison of the needs of the three age groups for various items in the section of cultural and recreational activities.

From Figure 16, it is not difficult to find that the elderly people aged 60–70 have a relatively high demand for health lectures. The need for sports is more obvious among the 70–80-year-olds. Similarly, the needs of the elderly over 80 years old are also concentrated in health lectures.

The reasons for this phenomenon are as follows: with the improvement of living standards, the elderly regardless of age group are paying more and more attention to health. For the health of the elderly over 80 years old, the focus is on treatment. In addition to the conventional treatment provided by the hospital, the elderly also want to find a way to assist the treatment in their daily life. Health lectures are also one of the ways to acquire such knowledge. For the elderly between the ages of 70 and 80, although the body is uncomfortable, it does not affect the quality of life. They prefer to improve their physical fitness and enrich their lives through appropriate physical exercise [23].

According to the above analysis, the summary is as follows: the elderly with different educational backgrounds have different needs for the elderly care services in smart communities. The higher the education level, the higher the demand for cultural entertainment and spiritual escort. This requires the community-based smart elderly care service platform conduct research on the needs of the elderly. Using the Internet and big data to provide the elderly with suitable elderly care services, there are also some direct or indirect problems in the entire service system. First of all, the professionalism of smart community elderly care service personnel is insufficient, and there is a lack of unified standards. Because the state has not issued a unified standard for the evaluation of practitioners, the professional quality of service personnel varies. Secondly, the classification of elderly care service levels is not clear, so that the elderly cannot get the appropriate elderly care services they want and dispel the enthusiasm of the elderly to accept, adapt, and participate. Finally, due to the lack of popularization of smart communities, the elderly do not have a clear understanding of the concept of smart community elderly care and the services included in smart elderly care [24]. Therefore, how to popularize the smart community pension and perfect it and do it better will make it easier for the elderly to understand and accept it.

## 6. Conclusions

Smart old-age care has greatly changed the traditional old-age care model and improved the quality of old-age care services. It can integrate government and community family resources, provide the most suitable way of old-age care for the elderly, and transfer old-age care from small homes to communities. Reducing the pressure of modern children will allow the elderly to get along well with the elderly and enjoy the life of the elderly themselves. While popularizing and developing smart elderly care services, the elderly are encouraged to treat the elderly kindly and participate in social activities, which is in line with the development of active aging.

## Figures and Tables

**Figure 1:** Human-computer interaction process based on somatosensory sensors.

**Figure 2:** Kinect for windows.

**Figure 3:** Kinect for Xbox.

**Figure 4:** API stack of Kinect SDK.

**Figure 5:** Leap motion somatosensory controller.

**Figure 6:** Target recognition and tracking process.

**Figure 7:** Finger kinematics model.

**Figure 8:** Overall architecture design diagram.

**Figure 9:** Technical architecture diagram of smart community elderly care service management system.

**Figure 10:** Functional architecture design of the smart community elderly care service management system.

**Figure 11:** Design diagram of basic data management function architecture.

**Figure 12:** Network architecture design diagram of smart community elderly care service management system.

**Figure 13:** Changes in the elderly population with household registration in a city from 2012 to 2017.

**Figure 14:** Function usage of smart elderly care platform for the elderly in a city.

**Figure 15:** Comparison of the demand for life services among the elderly in different age groups in a city.

**Figure 16:** Comparison of the demand for recreational activities among the elderly in different age groups in a city.

**Table 1:** Main technical specifications of Kinect.

Kinect features	Specifications
Effective sight distance	Default: 0.8–4.0, close-up mode 0.4–3.5
Viewing angle	43° vertically, 57° horizontally
Tilt range	±28°
Depth image	QVGA (320 *∗* 240)
Color image	VGA (640 *∗* 480)

**Table 2:** Histogram matching method reference table.

Match result	Related	Bangla	Intersect
Exact match	1.5	0.0	1.5
Half match	0.6	0.52	0.7
No match at all	−1.1	2.8	0.0

**Table 3:** User table.

Serial number	Meaning	Field	Types of	Size	Primary key
1	Serial number	User_Id	INT	25	Yes
2	Name	User_Name	VARCHAR	15	No
3	Community	Community	VARCHAR	100	Yes
4	Street	Street	VARCHAR	100	No
5	Category	Category	INT	3	No
6	Gender	Gender	INT	3	Yes
7	Date of birth	Date_Birth	DA TETIME	25	No
8	Condition	Status	INT	2	Yes
9	Home phone	Telephone	VARCHAR	20	Yes
10	Reviewer	Audit_Id	INT	25	No

**Table 4:** Service provider table.

Serial number	Meaning	Field	Type	Size	Primary key
1	Merchant coding	Business_Id	INT	25	No
2	The shop's name	Business_ Name	VARCHAR	45	No
3	Business category	Business_ Status	INT	10	Yes
4	Business license code	Business License_Code	VARCHAR	80	No
5	Service status	Service_Status	INT	1	Yes
6	Business hours	Business_ Hours	DATETIME	55	No
7	Principal	Principal	INT	45	No
8	Contact number	Contact Number	VARCHAR	20	No
9	Responsible area	Responsible_ Area	INT	55	No
10	Service personnel	Service_ Personnel	INT	50	No

**Table 5:** Activity sheet.

Serial number	Meaning	Field	Types	Size	Primary key
1	Event number	Activity_Id	INT	45	No
2	Event name	Activity_Name	VARCHAR	45	Yes
3	Type of activity	Activity_Type	VARCHAR	45	No
4	Hold time	Hold_ Time	DATETIME		Yes
5	Starting time	Starting _Time	DATETIME		No
6	End Time	End_ _Time	DATETIME		No
7	Event Location	Event_Location	VARCHAR	45	No
8	Next event	Next_ Event	DA TETIME		Yes
9	Contact number	Telephone	VARCHAR	20	Yes
10	Condition	Status	INT	2	No

**Table 6:** Service ticket form.

Serial number	Meaning	Field	Types of	Size	Primary key
1	Commodity code	Product_Id	INT	25	Yes
2	Product name	Product_ Name	VARCHAR	45	Yes
3	Specifications	Specification	DOUBLE	25	No
4	unit	Unit	VARCHAR	10	No
5	Number of Products	Quantity	INT	50	No
6	Commodity price	Unit_ Price	DOUBLE	25	Yes
7	Total price	Total Price	DOUBLE	25	Yes
8	Number Delivery	Number_ Delivery	VARCHAR	40	No
9	Old man's name	Elderly_ Name	VARCHAR	25	No
10	Elderly contact information	Elderly_ Tel	VARCHAR	50	Yes
11	Address	Elderly_ Address	VARCHAR	20	Yes
12	Payment method	Payment_ Method	VARCHAR	20	No

## Data Availability

Data sharing is not applicable to this article as no datasets were generated or analyzed during the current study.
